# Activation Studies of the β-Carbonic Anhydrase from the Pathogenic Protozoan *Entamoeba histolytica* with Amino Acids and Amines

**DOI:** 10.3390/metabo9020026

**Published:** 2019-02-01

**Authors:** Silvia Bua, Susanna Haapanen, Marianne Kuuslahti, Seppo Parkkila, Claudiu T. Supuran

**Affiliations:** 1 Sezione di Scienze Farmaceutiche e Nutraceutiche, Dipartimento Neurofarba, Università degli Studi di Firenze, Via U. Schiff 6, 50019 Sesto Fiorentino, 50019 Florence, Italy; silvia.bua@unifi.it; 2 Faculty of Medicine and Health Technology, Tampere University, 33100 Tampere, Finland; Haapanen.Susanna.E@student.uta.fi (S.H.); Marianne.Kuuslahti@staff.uta.fi (M.K.); seppo.parkkila@staff.uta.fi (S.P.); 3 Fimlab Ltd., Tampere University Hospital, 33100 Tampere, Finland

**Keywords:** *Entamoeba histolytica*, carbonic anhydrase, metalloenzymes, protozoan, amine, amino acid, activator

## Abstract

The β-carbonic anhydrase (CA, EC 4.2.1.1) from the pathogenic protozoan *Entamoeba histolytica*, EhiCA, was investigated for its activation with a panel of natural and non-natural amino acids and amines. EhiCA was potently activated by D-His, D-Phe, D-DOPA, L- and D-Trp, L- and D-Tyr, 4-amino-L-Tyr, histamine and serotonin, with K_A_s ranging between 1.07 and 10.1 µM. The best activator was D-Tyr (K_A_ of 1.07 µM). L-Phe, L-DOPA, L-adrenaline, L-Asn, L-Asp, L-Glu and L-Gln showed medium potency activation, with K_A_s of 16.5–25.6 µM. Some heterocyclic- alkyl amines, such as 2-pyridyl-methyl/ethyl-amine and 4-(2-aminoethyl)-morpholine, were devoid of EhiCA activating properties with K_A_s > 100 µM. As CA activators have poorly been investigated for their interaction with protozoan CAs, our study may be relevant for an improved understanding of the role of this enzyme in the life cycle of *E*. *histolytica*.

## 1. Introduction

Recently, we have reported [1,2] the cloning, purification and characterization of a β-carbonic anhydrase (CA, EC 4.2.1.1) present in the genome of the pathogenic protozoan *Entamoeba histolytica*, the etiological agents provoking amebiasis, an endemic disease in developing countries and also affecting travelers returning from risk zones [3,4,5]. In addition, invasive forms of *E. histolytica* infection were reported to lead to liver cysts, associated frequently with complications such as pleural effusion due to the rupture of the cysts as well as dissemination to extra-intestinal organs, e.g., the brain or pericardium, which occasionally may have fatal consequences [3,6]. In the previous work [1,2] we also investigated the inhibition profile of the new enzyme (nominated EhiCA) with the main classes of CA inhibitors (CAIs) [7,8,9,10], the sulfonamides and the inorganic anions [11,12,13,14]. Our main scope was to identify agents that by interference with the activity of this enzyme, might lead to anti-infectives with a novel mechanism of action, considering the fact that many CAs are essential in the life cycle of microorganisms belonging to the bacteria, fungal or protozoan domains [15,16,17]. As β-CAs are not present in mammals [18,19], effective EhiCA inhibitors may represent an alternative therapeutic option for this protozoan infection. In fact, in the previous work we have shown that inhibition of other protozoan CAs, such as the β-class enzyme from *Leishmania donovani* [20,21] or the α-CA from *Trypanosoma cruzi* [20,22,23], has important antiparasitic effects in vitro and in vivo [21].

Indeed, various pathogenic organisms belonging to the bacteria, fungal or protozoan domains encode for CAs, which have been investigated in some detail ultimately, in the search of anti-infectives with a diverse mechanism of action [7,8,9,10,14,15,16,17,18,19,20,21,22,23]. CAs catalyze the reaction between CO_2_ and water, with formation of bicarbonate (HCO_3_^-^) and protons (H^+^), and are highly effective catalysts, among the most efficient known so far in nature [7,8,9,10]. CAs are involved in various biochemical and metabolic processes, among which are acid-base homeostasis, respiration, biosynthesis of various metabolites (urea, glucose, fatty acids, carbamoyl phosphate), electrolytes secretion, etc. [7,8,9,10,11,12]. Seven distinct CA families are known to date, the α, β, γ, δ, ζ, ƞ and θ class CAs, which are widespread all over the phylogenetic tree, from simple organisms, such as bacteria and Archaea, to more complex ones, such as vertebrates [7,8,9,10,24,25,26,27,28]. These diverse CA genetic families do not share significant sequence homology or structural identity, being an interesting example of convergent evolution at the molecular level [7,8,9,10]. In humans, as in many other vertebrates, only α-CAs are present, and their inhibition has been exploited from the pharmacological viewpoint for decades, for drugs such as diuretics [29], anticonvulsants [29,30], antiobesity [30] and more recently, antitumor agents [31]. However, these enzymes may also be activated [32] but the CA activators (CAAs) have seen fewer applications up until now. However, recent studies [33] pointed out to the possible application of CAAs targeting human enzymes for the enhancement of cognition. The nonvertebrate CAs were on the other hand only in the last few years investigated in some detail [34,35,36,37]. Here we report the first activation study of the β-CA from *E. histolytica* with a panel of amines and amino acid derivatives. As CAAs have poorly been investigated for their interaction with protozoan CAs, our study may be relevant for an improved understanding of the role of this enzyme in the life cycle of *E. histolytica*.

## 2. Results and Discussion

The catalytic activity of the recombinant EhiCA (for the CO_2_ hydration reaction), has been recently reported [1,2], being measured by using a stopped flow technique [38]. EhiCA showed a significant catalytic activity for the physiologic, CO_2_ hydration reaction, with the following kinetic parameters: k_cat_ = 6.7 × 10^5^ s^−1^ and k_cat_/K_m_ = 8.9 × 10^7^ M^−1^ × s^−1^. Thus, EhiCA is 1.8 times more effective as a catalyst compared to the slow human (h) isoform hCA I (considering the k_cat_/K_m_ values) or 3.35 times more effective than hCA I (considering only the kinetic constant k_cat_) [1,2]. EhiCA activity was also inhibited by the standard, clinically used sulfonamide CA inhibitor acetazolamide (AZA, 5-acetamido-1,3,4-thiadiazole-2-sulfonamide), with a K_I_ of 509 nM (data not shown here) [1,2].

Similar to all β-CAs investigated to date, EhiCA has a catalytically crucial zinc ion and its conserved protein ligands, which for this enzyme are: Cys50, His103 and Cys106 [1,2]. The fourth metal ion ligand is a water molecule/hydroxide ion, which acts as nucleophile in the catalytic cycle (Equation (1) below). A catalytic dyad constituted by the pair Asp52-Arg54 [1,2], conserved in all enzymes belonging to the β-class is also present in EhiCA, presumably with the role to enhance the nucleophilicity of the zinc-coordinated water molecule [18,19,20]. However, the rate-determining step for many CAs is the generation of the nucleophilic species of the enzyme, represented by Equation (2) below:

H_2_O

EZn^2+^—OH^−^ + CO_2_ ⇔ EZn^2+^—HCO_3_^-^ ⇔ EZn^2+^—OH_2_ + HCO_3_ (1)

EZn^2+^— -OH_2_ ⇔ EZn^2+^—OH^−^ + H^+^ (2)

In most CAs, this step (Equation (2)) is assisted by amino acid residues from the active site [32], becoming an intramolecular step (instead of an intermolecular one), which is favored thermodynamically. Furthermore, the activators (CAAs) may participate in this step, as outlined in Equation (3):

EZn^2+^— -OH_2_ + A ⇔ [EZn^2+^— -OH_2_ − A] ⇔ [EZn^2+^—OH^−^ − AH^+^] ⇔ EZn^2+^—OH^−^ + AH^+^ (3)

enzyme - activator complexes

The enzyme forms with the activator complexes (E-A complexes, where E stands for enzyme and A for activator), in which the proton transfer step from the zinc-coordinated water to the environment is intramolecular and thus, more efficient than the corresponding intermolecular process shown schematically in Equation (2) [32]. In fact, X-ray crystal structures are available for many CAs to which activators are bound within the active site [32,39,40,41], but only for α-class enzymes these structures have been reported to date. The activator binding site for the α-CAs is situated at the entrance of the active site cavity not far away from His64, which acts as proton shuttle residue in the process described by Equation (2) [32,39,40,41].

We have performed detailed kinetic measurements of EhiCA activity in the presence of amine and amino acid activators (Figure 1), such as for example L-Trp (Table 1). Data of Table 1 show that the presence of L-Trp does not change the K_M_, both for the α-class enzymes hCA I/II as well as the β-CA, EhiCA, investigated here. Interestingly, it has an effect on the k_cat_, which at 10-µM concentration of activator leads to a 2.83 times enhancement of the kinetic constant for the protozoan enzyme, from 6.7 × 10^5^ s^−1^ to 1.9 × 10^6^ s^−1^ (Table 1).

In order to obtain an activation profile of EhiCA with a wide range of amino acid and amine activators of types 11–24, we performed dose response curves of the activation of EhiCA in the presence of increasing concentrations of activators, in order to determine the activation constants K_A_-s (see Materials and Methods for details). We included in our study the amino acids and amines which were investigated as activators of CAs belonging to various classes from diverse organisms [32,33,34,35,36,37,40,41,42]. These activation data are reported in Table 2, in which, for comparison reasons, the activation of the human isoforms hCA I and II and of the protozoan β-CA from *Leishmania donovani chagasi* are also presented.

The structure–activity relationship (SAR) for the activation of EhiCA with compounds **1**–**24** revealed the following observations:

(i) Some heterocyclic-alkyl amines, such as 2-pyridyl-methyl/ethyl-amine **15**, **16** and 4-(2-aminoethyl)-morpholine, were devoid of EhiCA activating properties up to 100 µM concentration of activator in the assay system. All these compounds are structurally related, possessing a heterocyclic ring and aminomethyl/aminoethyl moieties in their molecules.
(ii) L-His, dopamine, 1-(2-aminoethyl)-piperazine and D-Glu were poor EhiCA activators, with activation constants ranging between 30.3 and 78.7 µM (Table 2). There is no strong structural correlation between these three compounds.
(iii) Many of the compounds investigated here showed medium potency efficacy as EhiCA activators, with K_A_s ranging between 16.5 and 25.6 µM. They include L-Phe, L-DOPA, L-adrenaline, L-Asn, L-Asp, L-Glu and L-Gln. It may be observed that there are no remarkable differences of activity between the pairs L-Asp/L-Asn and L-Glu/L-Gln, whereas D-Glu was more ineffective compared to L-Glu. This is in fact the exception, as for other L-/D-enantiomeric amino acids investigated here, the D-enantiomer was the most effective activator (see later in the text).
(iv) Effective EhiCA activating properties were detected for the following amino acids/amines: D-His, D-Phe, D-DOPA, L- and D-Trp, L- and D-Tyr, 4-amino-L-Tyr, histamine and serotonin, which showed K_A_s ranging between 1.07 and 10.1 µM. The best activator was D-Tyr (K_A_ of 1.07 µM). In fact for all aromatic amino acids investigated here, the D-enantiomer was more effective as EhiCA activator compared to the corresponding L-enantiomer. For the Phe-Tyr-DOPA subseries, the activity increased by hydroxylation of the Phe, achieving a maximum for Tyr and then slightly decreased with the introduction of an additional OH moiety in DOPA, but always the D-enantiomers were better activators compared to the L-ones. The loss of the carboxyl moiety, such as in histamine and serotonin, did not lead to important changes of activity compared to the corresponding D-amino acids, but in the case of dopamine, the activating efficacy was much lower compared to those of both L- and D-DOPA.
(v) The activation profile of EhiCA with amino acid and amine derivatives is rather different from those of other CAs, among which the protozoan β-CA from *Leishmania donovani chagasi* (LdcCA) or the α-class human CAs, isoforms hCA I and II. For example **17** was a nanomolar activator for LdcCA whereas its affinity for EhiCA was of only 43.8 µM. For the moment, no EhiCA-selective activators were detected.

## 3. Materials and Methods

### 3.1. EhiCA Production and Purification

The protocol described in [1,2] has been used to obtain purified recombinant EhiCA. All activators were commercially available from Sigma-Aldrich (Milan, Italy) and were of the highest purity available.

### 3.2. CA activity and Activation Measurements

An Sx.18Mv-R Applied Photophysics (Oxford, UK) stopped-flow instrument has been used to assay the catalytic activity of various CA isozymes for CO_2_ hydration reaction [38]. Phenol red (at a concentration of 0.2 mM) was used as indicator, working at the absorbance maximum of 557 nm, with 10 mM Hepes (pH 7.5, for α-CAs) or TRIS (pH 8.3, for β-CAs) as buffers, 0.1 M NaClO_4_ (for maintaining constant ionic strength), following the CA-catalyzed CO_2_ hydration reaction for a period of 10 s at 25 °C. The CO_2_ concentrations ranged from 1.7 to 17 mM for the determination of the kinetic parameters and inhibition constants. For each activator at least six traces of the initial 5–10% of the reaction have been used for determining the initial velocity. The uncatalyzed rates were determined in the same manner and subtracted from the total observed rates. Stock solutions of activators (at 0.1 mM) were prepared in distilled-deionized water and dilutions up to 1 nM were made thereafter with the assay buffer. Enzyme and activator solutions were pre-incubated together for 15 min prior to assay, in order to allow for the formation of the enzyme–activator complexes. The activation constant (K_A_), defined similarly with the inhibition constant K_I_, can be obtained by considering the classical Michaelis–Menten equation (Equation (4)), which has been fitted by nonlinear least squares by using PRISM 3:

v = v_max_/{1 + (K_M_/[S]) (1 + [A]_f_/K_A_)} (4)

where [A]_f_ is the free concentration of activator.

Working at substrate concentrations considerably lower than K_M_ ([S] << K_M_), and considering that [A]_f_ can be represented in the form of the total concentration of the enzyme ([E]_t_) and activator ([A]_t_), the obtained competitive steady-state equation for determining the activation constant is given by Equation (5):

v = v_0_ · K_A_/{K_A_ + ([A]_t_ − 0.5{([A]_t_ + [E]_t_ + K_A_) − ([A]_t_ + [E]_t_ + K_A_)^2^ − 4[A]_t_ · [E]_t_)^1/2^}} (5)

where v_0_ represents the initial velocity of the enzyme-catalyzed reaction in the absence of activator [32,41,42].

## 4. Conclusions

We report the first activation study of the β-CA from the protozoan parasite *Entamoeba histolytica*, EhiCA, with a panel of amino acids and amines, some of which are important autacoids. The enzyme was potently activated by D-His, D-Phe, D-DOPA, L- and D-Trp, L- and D-Tyr, 4-amino-L-Tyr, histamine and serotonin, with K_A_s ranging between 1.07 and 10.1 µM. The best activator was D-Tyr (K_A_ of 1.07 µM). L-Phe, L-DOPA, L-adrenaline, L-Asn, L-Asp, L-Glu and L-Gln showed medium potency activation, with K_A_s of 16.5–25.6 µM. Some heterocyclic-alkyl amines, such as 2-pyridyl-methyl/ethyl-amine and 4-(2-aminoethyl)-morpholine, were devoid of EhiCA activating properties with K_A_s > 100 µM. The X-ray crystal structure of this enzyme is not known for the moment, and in addition, no adducts of other parasite enzymes complexed with activators are available so far in order to rationalize our results. However, as CAAs have poorly been investigated for their interaction with protozoan CAs, our study may be relevant for an improved understanding of the role of this enzyme in the life cycle of *E. histolytica*.

## Figures and Tables

**Figure 1:** CAAs of type **1–24** used in the present study.

**Table 1:** Activation of human carbonic anhydrase (hCA) isozymes I, II, and EhiCA with L-Trp at 25 °C for the CO_2_ hydration reaction [38].

Isozyme	k_cat_ *	K_M_ *	(k_cat_)_L-Trp_ **	K_A_ *** (µM)
	(s^−1^)	(mM)	(s^−1^)	L-Trp
hCA I ^a^	2.0 × 10^5^	4.0	3.4 × 10^5^	44.0
hCA II ^a^	1.4 × 10^6^	9.3	4.9 × 10^6^	27.0
LdCA	9.35 × 10^5^	15.8	1.9 × 10^6^	4.02
EhiCA ^b^	6.7 × 10^5^	7.5	1.9 × 10^6^	5.24

* Observed catalytic rate without activator. K_M_ values in the presence and the absence of activators were the same for the various CAs (data not shown).; ** Observed catalytic rate in the presence of 10 µM activator; *** The activation constant (K_A_) for each enzyme was obtained by fitting the observed catalytic enhancements as a function of the activator concentration [41]. Mean from at least three determinations by a stopped-flow, CO_2_ hydrase method [38]. Standard errors were in the range of 5–10% of the reported values (data not shown); ^a^ Human recombinant isozymes, from ref. [32]; ^b^ Protozoan recombinant enzyme, this work.

**Table 2:** Activation constants of hCA I, hCA II and the protozoan enzymes LdcCA (*L. donovani chagasi*) and EhiCA (*E. histolytica*) with amino acids and amines **1**–**24**. Data for hCA I and II are from [32] and for LdcCA from [42].

No.	Compound		K_A_ (mM) *		
		**hCA I ^a^**	**hCA II ^a^**	**LdcCA ^b^**	**EhiCA ^c^**
**1**	L-His	0.03	10.9	8.21	78.7
**2**	D-His	0.09	43	4.13	9.83
**3**	L-Phe	0.07	0.013	9.16	16.5
**4**	D-Phe	86	0.035	3.95	10.1
**5**	L-DOPA	3.1	11.4	1.64	16.6
**6**	D-DOPA	4.9	7.8	5.47	4.05
**7**	L-Trp	44	27	4.02	5.24
**8**	D-Trp	41	12	6.18	4.95
**9**	L-Tyr	0.02	0.011	8.05	4.52
**10**	D-Tyr	0.04	0.013	1.27	1.07
**11**	4-H_2_N-L-Phe	0.24	0.15	15.9	8.12
**12**	Histamine	2.1	125	0.74	7.38
**13**	Dopamine	13.5	9.2	0.81	30.8
**14**	Serotonin	45	50	0.62	4.94
**15**	2-Pyridyl-methylamine	26	34	0.23	>100
**16**	2-(2-Aminoethyl)pyridine	13	15	0.012	>100
**17**	1-(2-Aminoethyl)-piperazine	7.4	2.3	0.009	43.8
**18**	4-(2-Aminoethyl)-morpholine	0.14	0.19	0.94	>100
**19**	L-Adrenaline	0.09	96	4.89	25.6
**20**	L-Asn	11.3	>100	4.76	23.8
**21**	L-Asp	5.2	>100	0.3	23.9
**22**	L-Glu	6.43	>100	12.9	25.5
**23**	D-Glu	10.7	>100	0.082	30.3
**24**	L-Gln	>100	>50	2.51	20.1

* Mean from three determinations by a stopped-flow, CO_2_ hydrase method [38]. Standard errors were in the range of 5–10% of the reported values (data not shown). ^a^ Human recombinant isozymes, from ref. [32]; ^b^ Protozoan recombinant enzyme, from ref. [42]; ^c^ This work.
